The article "Manifestation of Urinary Tract Injury during Cervical Cancer Surgery Based on CT Urography Secretion Phase Images" was published in 2022. Journal: Contrast Media Mol Imaging.

# Manifestation of Urinary Tract Injury during Cervical Cancer Surgery Based on CT Urography Secretion Phase Images

**DOI:** 10.1155/2022/2572681

**Published:** 2022-06-15

**Authors:** Song Lin, Xiaoshan Li, Yan Zhang, Xiaowen Mao, Xingchi Liang, Shigang Cheng, Lingli Zhang

**Affiliations:** ^1^Department of Surgery, Maternal and Child Health Hospital of Hubei Province, Wuhan 430070, Hubei, China; ^2^Department of Urology, Yangtze River Shipping General Hospital, Wuhan 430014, Hubei, China; ^3^Department of Women's Health, Maternal and Child Health Hospital of Hubei Province, Wuhan 430070, Hubei, China; ^4^Department of Gynecology, Maternal and Child Health Hospital of Hubei Province, Wuhan 430070, Hubei, China

## Abstract

**Methods:**

We grouped the patients who had undergone cervical cancer surgery in a hospital in this article and compared the nanodrug carrier system under CT imaging with traditional laparoscopy. The postoperative physical parameters of surgical patients are collected from cervical cancer patients of different degrees, and the parameters and prognostic health of patients after different operations are compared.

**Results:**

The results of the study show that the postoperative patient's body parameters of the nanodrug delivery system under the CT imaging technology used in this article are better than those of the traditional surgery group, and the average intraoperative blood loss is about 20% less than that of the traditional surgery. Postoperative complications occur. The situation is even lower, more than 30% lower than traditional surgery.

**Conclusion:**

This shows that the operation of the nanodrug delivery system based on CT imaging technology has broken through some of the limitations of the development of laparoscopic technology and has played an important role in the surgical treatment of cervical cancer.

## 1. Introduction 

Cervical cancer is often referred to as cervical cancer. These are the three most common malignant tumors in the female genital system. In recent years, cervical smear specimens have been widely used, and early detection and treatment of cervical cancer and precancerous lesions have greatly reduced the infection rate and mortality rate [1]. However, in China, the incidence of cervical cancer is still at the forefront of the incidence of female malignant tumors and cervical cancer. The uterus tends to be younger, which is one of the malignant tumors that must be considered in the prevention and treatment of cancer. According to the World Health Organization, Chile, China, and Venezuela have the highest incidence of cervical cancer in the world. More than 85% of diseases occur in developing countries, accounting for 13% of all women suffering from cancer. Cervical cancer patients are mainly distributed in the central and western regions, and the rural areas are slightly higher than those in the cities. The incidence of cervical cancer varies greatly geographically. The incidence of cervical cancer is also related to economic development.

The article "Manifestation of Urinary Tract Injury during Cervical Cancer Surgery Based on CT Urography Secretion Phase Images" was published in 2022. Journal: Contrast Media Mol Imaging.

The treatment methods of cervical cancer mainly include comprehensive treatment methods such as surgery, radiation therapy, and chemotherapy. Although treatment methods such as radiotherapy and traditional chemotherapy continue to improve, surgery is still the first choice for the treatment of early-stage cervical cancer. The surgical treatment of cervical cancer includes laparotomy, laparoscopic surgery, and robotic laparoscopic surgery. In recent years, with the use of many new technologies and new machines, the surgical methods of cervical cancer have also undergone great changes in clinical diagnosis and treatment [2]. The circulation of nanomedium refers to the use of nanomaterial technology to form a nanomedium circulation system through drugs and carriers (including inorganic materials and polymer materials). The nanodrug carrier contains trees, fungi, nanotorrents, and inorganic nanoparticles. Generally speaking, anticancer agents are small hydrophobic molecules, which are difficult to absorb directly from the body. In order to improve the water solubility and stability of the drug, reduce side effects, expand the effective treatment level of the drug, improve the effectiveness and use rate, and finally achieve the purpose of inhibiting the proliferation and spread of tumor cells, the anticancer agent can be used for diffusion adsorption, inoculation, and association. Methods such as shaft devices are integrated into the nanomedia system. In terms of the development and design of pharmaceutical companies, pharmaceutical companies are getting more and more attention.

Regarding the issue of cervical cancer, experts at home and abroad have also conducted many studies. Luvero et al. used single-factor and multifactor analysis to analyze the prognostic factors that may affect survival more in the long term. In this study, we included all patients diagnosed with locally advanced cervical cancer (IB2-IIB) in June 2000 and February 2007, as described by Angioli et al. (Gynecol Oncol 127(2):290–62012). The primary endpoint of the study is the overall survival (OS) of patients with lymph node metastasis and patients without lymph node positive at the end of the 10-year follow-up to confirm the impact of lymph node metastasis on long-term prognosis. In addition, we also analyzed other factors that affect the prognosis, such as tissue type, tumor size, grade, and paracancerous invasion [3]. Smith et al. determined the incidence and risk factor of parameterized intervention (PI) based on cone specimens (CS) and potentially identified candidate factors for less radical surgery. Retrospective analysis of the clinical data of FIGO IA2-IIA cervical cancer treated by radical hysterectomy and pelvic lymph node dissection (RH) from 2000 to 2010. The information is taken from the surgical and pathological reports. Fisher's exact test, *t*-test, and asymptotic logistic regression were used for statistical analysis. Of the 267 RH patients, 118 (44%) underwent conization before RH. Before RH, the incidence of PI after conization treatment was 15.7% and 7.5%. PI has no correlation with histology, staging, grade, or tumor size [4]. Peng et al. evaluated the efficacy and safety of neoadjuvant chemotherapy (NACT) and radical surgery (RS) in the treatment of cervical cancer. A meta-analysis of randomized controlled trials (RCT) between NACT + RS and RS alone in cervical cancer patients was carried out according to the guidelines for the preferred reporting items of systematic reviews and meta-analysis (PRISMA) reports. From the establishment to April 2015, the following electronic databases and Cochrane libraries were searched. We use REVIEW MANAGER 5.3 for statistical analysis. Five randomized controlled trials were conducted on 739 patients. The results showed that there was a significant difference in the positive rate of lymph nodes between the NACT + RS group and the RS group alone [5]. Liu et al. analyzed the curative effect and adverse reactions of postoperative radiotherapy in 98 cases of stage I∼III cervical cancer. From 2006 to 2014, 98 patients with stage I-III cervical cancer received postoperative radiotherapy. The histological type was mainly squamous cell carcinoma, accounting for 92.86% (91 cases). Postoperative radiotherapy methods included two-field radiation (16 cases, 16.32%), four-field box radiation (16 cases, 16.32%), and intensity-modulated radiotherapy (IMRT) (66 cases, 67.36%)). The survival rate was expressed by Kaplan–Meier curve, and the prognostic analysis was analyzed by Cox multivariate analysis. The 5-year overall survival rate and progression-free survival rate were 82.0% and 76.0%, respectively [6]. These studies have provided some references for this article, but due to insufficient research samples, there is a little doubt about the validity of the data, leading to some problems with the conclusions of these studies.

The article "Manifestation of Urinary Tract Injury during Cervical Cancer Surgery Based on CT Urography Secretion Phase Images" was published in 2022. Journal: Contrast Media Mol Imaging.

Compared with traditional cervical cancer treatment methods, this article creatively uses nanodrug delivery system to study the urinary tract injury during cervical cancer surgery and proves that the nanodrug delivery system slowly releases drugs in response to the stimulation of the cancer tissue microenvironment and can achieve treatment. The effect of cancer, a comprehensive clinical analysis of the case materials of urinary tract injuries during and after surgery, studies the related factors of urinary tract injury in the treatment of cervical cancer, achieves early detection and timely treatment of urinary tract injuries, and maintains a high degree of urinary system protection and injury prevention awareness, which actively take preventive measures, try to avoid iatrogenic injury, and improve the treatment effect and prognosis of patients.

## 2. Methods of Research on the Impact of Urinary Tract Injury during Cervical Cancer Surgery

### 2.1. CT Imaging Treatment

CT is based on the difference in the degree of absorption of X-rays by the detected object. The X-ray is converted into visible light by the detector, and then, this visible light is converted into an electrical signal, which is then converted into a signal that can be processed by a computer system by an analog/digital converter. After computer processing, the X-ray absorption coefficient of each voxel can be obtained by calculation, which is arranged in a digital matrix. Then, the digital/analog converter converts the elements at each position in these digital matrices into small blocks with different gray levels that gradually decrease in brightness from black to white, called pixels, and press these small blocks with different gray levels. Finally, matrix arrangement gets the CT image.

Because X-rays can penetrate metal materials, there is a metal end cap for fixing concrete specimens in this test, so it is appropriate to use X-CT technology for this test. When X-rays penetrate an object, different materials absorb X-rays in different degrees, resulting in different gray values of each material, and different gray values form the final CT image.

Nanomedical institutions have a wide range of materials and manufacturing methods, including nanoliposomes, nanomixtures, nanoparticles, and dendritic particles [7, 8]. With the continuous development of biomedical materials and the continuous improvement of human living standards, more and more nanopharmaceutical carriers have been designed, and they must meet the safety, intelligence, and protection of drugs in the body. The normal characteristics of carcinogenic tissues form the basis for the design of these vectors [9].

The normal characteristics of tissue volume constitute the basis for the construction of nanomedicine carriers. The influence of tissue volume on nanoparticles, with the unlimited proliferation of cancer cells, the number of blood vessels, and lymph nodes in cancer tissues, continues to increase, but the pores in the new blood vessels are very large. Nanoparticles of a certain size will increase tumor invasion and decrease [10]. This is why nanomedical institutions can target tumor tissues and accumulate in lesions [11]. This is the increasing intelligence of medical institutions with pH targeting functions. The basis of the drug delivery system with little or no expression in normal tissues is shown in Figure 1.

The article "Manifestation of Urinary Tract Injury during Cervical Cancer Surgery Based on CT Urography Secretion Phase Images" was published in 2022. Journal: Contrast Media Mol Imaging.

With the development of materials science, biomedicine, and clinical science, drug carriers have become an emerging research content, and the design requirements of drug carriers have also been continuously improved. The drug carrier can protect the drug from the physiological environment, improve the stability of the drug, and reduce the toxic and side effects of the drug on the organism [12]. The drug carrier can also make the release mode, rate, and location of the drug selective and controllable. The construction of a targeted nanodrug delivery system is of great significance in biomedicine. It can control the selectivity, rate, and form of drug release, and at the same time, it can improve the stability of the drug and reduce the toxic and side effects of the drug on the organism.

### 2.2. Cervical Cancer

At present, the cause of cervical cancer is unclear. Epidemiological studies have found that cervical cancer is related to human mammary virus (HPV) infection, precocious puberty, multiple sexual partners, sexual dysfunction, sexually transmitted diseases, smoking, low economic status, and immunosuppression. Ion infection is a persistent infection of high-risk human mammalian virus (HPV), which is the main risk factor [13]. More than 95% of cervical cancers are accompanied by high-risk HPV infections. Uterine laryngeal cancers caused by types 16 and 18 account for about 70% of cervical cancers [14].

The staging of cervical cancer is clinical staging, using the International Union of Obstetrics and Gynecology (FIGO) staging standards, as shown in Table 1.

The treatment methods of cervical cancer mainly include comprehensive treatments such as surgery, radiotherapy, and chemotherapy. Despite the continuous improvement of treatment methods such as radiotherapy and conventional chemotherapy, surgery is still the first choice for the treatment of early cervical cancer [15, 16]. The surgical treatment of cervical cancer includes open surgery, laparoscopic surgery, and robotic laparoscopic surgery. In recent years, with the continuous application of new technologies and equipment, the surgical methods for cervical cancer have also undergone tremendous changes in clinical practice. In recent years, nanomedicine delivery systems for the treatment of gynecological malignant tumors have also received more and more clinical applications in my country, and have developed into a new level [17]. The treatment process is shown in Figure 2.

The article "Manifestation of Urinary Tract Injury during Cervical Cancer Surgery Based on CT Urography Secretion Phase Images" was published in 2022. Journal: Contrast Media Mol Imaging.

At present, the surgical operation of the nanodrug delivery system still belongs to laparoscopic surgery. Therefore, in addition to inheriting the advantages of minimally invasive laparoscopic surgery, it has some unique advantages [18]. The terminal organs of the nanodrug surgery system have multiple functions, allowing the operator performs complex surgical operations in a small space. In addition, the surgical operation of the nanodrug delivery system reduces the number of people involved in the operation, and the surgeon may need more time to occasionally stop for the operation, reduce fatigue, and be able to collect more energy to complete the long and complicated operation. From the patient's point of view, surgical operations are more accurate, reducing tissue trauma during the operation, reducing blood loss, and improving the accuracy and success of the operation [19]. The postoperative recovery is fast, the healing is good, the cosmetic effect is good, and the wound is small. We reduce postoperative pain and postoperative congestion.

Surgical nanodrug distribution systems have surpassed some of the limitations of the development of laparoscopic technology. This is a new technique for minimally invasive surgery. It has many advantages, provides convenience for gynecological tumor patients, and has good application prospects in gynecological surgery [20, 21]. With its further development, it is expected to overcome its shortcomings in the future, such as long preoperative preparation work, large equipment, complex installation, and high cost.

### 2.3. Medical Image Enhancement

Image enhancement is to highlight some information in the image, while removing or reducing some unwanted information. Image enhancement includes spatial enhancement and frequency enhancement [22]. Spatial enhancement is achieved through grayscale mapping transformation in the spatial domain, for example, histogram equalization. Frequency domain enhancement is to modify the corresponding frequency components in the frequency domain to achieve an enhancement effect, for example, changing the low-frequency area to smooth the image and changing the high-frequency area to sharpen the image [23]. This article uses the airspace enhancement method to process the patient's urinary tract image, and the formula is as follows:

(1) $$\begin{array}{c} g\left(x,y\right)=T\left[f\left(x,y\right)\right]. \end{array}$$

Among them, *f*(*x*, *y*) represents the input, *T* represents the mapping transformation function, and *g*(*x*, *y*) represents the output.

The article "Manifestation of Urinary Tract Injury during Cervical Cancer Surgery Based on CT Urography Secretion Phase Images" was published in 2022. Journal: Contrast Media Mol Imaging.

Histogram transformation is to enlarge the spacing of the gray value of the image, so that the dynamic range of the image becomes larger, and the details become more delicate and clear, so as to highlight the target information and facilitate observation. For an input image, *f*(*x*, *y*) grayscale histogram is as follows:

(2) $$\begin{array}{c} P_{r}\left(r_{k}\right)=\frac{n_{k}}{n}\;k=0,1,\ldots ,L-1. \end{array}$$

Among them, *L* represents the gray value range, *n* represents the total number of pixels, and *n*_*k*_ represents the number of pixels with a gray value of *k*. Through the above conditions, we can be drawn

(3) $$\begin{array}{c} P_{s}\left(s\right)=P_{r}\left|r\right|\frac{ds}{da}. \end{array}$$

The gray value of an image can be expressed as a random variable in the interval [0, 1]. The probability density function is one of the most basic descriptions of random variables, which can be obtained

(4) $$\begin{array}{c} ds=\frac{p_{r}\left(r\right)da}{P_{a}\left(a\right)}=\frac{p_{r}\left(r\right)da}{1}=P_{r}\left(r\right)dr. \end{array}$$

Thereby,

(5) $$\begin{array}{c} s=T\left(r\right)=\int_{0}^{r}P_{r}\left(s\right)\text{d}a. \end{array}$$

Among them, *T*(*r*)=*n*!/*r*!(*n* − *r*)! is the cumulative distribution function, and the digitized formula for the uniform distribution of the histogram is as follows:

(6) $$\begin{array}{c} s_{k}=T\left(r_{k}\right)=\sum_{i=0}^{k}P\left(r_{j}\right)=\sum_{j=0}^{k}\frac{n_{j}}{n}. \end{array}$$

We assign the *s*_*k*_ calculated in the formula to each quantization level according to a fixed interval

(7) $$\begin{array}{c} l_{k}=\left[s_{k}\left(L-1\right)\right]. \end{array}$$

In order to enhance the gray level of the target area information of different images, it is necessary to transform the histogram of the input image into some specific shapes. Therefore, the enhancement method of the histogram specification is obtained. The basic idea of prescribing is to transform the histogram of the input image to obtain a histogram of a specific shape for specific enhancement. The algorithm principle is as follows:

First, we perform histogram equalization

(8) $$\begin{array}{c} s_{k}=T\left(rk\right)=\sum_{j=1}^{k}p_{r}\left(r_{j}\right)=\sum_{j=1}^{k}\frac{ni}{n}. \end{array}$$

Then, we target image equalization

(9) $$\begin{array}{c} v_{x}=F\left(z_{k}\right)=\sum_{i=1}^{k}p_{z}\left(z_{i}\right),\;k=0,1,2,\ldots ,L-1. \end{array}$$

At this time, the uniformity of the two images is the same, that is, *v*_*x*_=*s*_*k*_, take the inverse transformation, and then substitute it into sk to get the specific gray level required

(10) $$\begin{array}{c} Z_{k}=G^{-1}\left(v_{k}\right)=G^{-1}\left(s_{k}\right). \end{array}$$

The image is subject to external and internal interference during the acquisition and preprocessing, resulting in some noise. Noise will degrade the image quality and affect the subsequent image processing results. Therefore, this paper uses adaptive median filtering and Wiener filtering to remove these noises. The traditional median filter formula is as follows:

(11) $$\begin{array}{c} g\left(x,y\right)=\text{med}\left\{f\left(x-k,y-1\right),\left(k,l\right)\in S\right\}. \end{array}$$

Among them, *f*(*x*, *y*) represents the input image, *S* represents the neighborhood (*x*, *y*) filter window of the pixel, and *g*(*x*, *y*) represents the output response. We calculate the local mean and variance of each pixel

(12) $$\begin{array}{c} \mu =\frac{1}{MN}\sum_{\left(n_{1},n_{2}\right)\in \mu }g\left(n_{1},n_{2}\right),\\ \sigma^{2}=\frac{1}{MN}{\sum_{\left(n_{1},n_{2}\right)\in \kappa }\left[g\left(n_{1},n_{2}\right)-\kappa \right]}^{2}. \end{array}$$

According to the characteristics of the image, the histogram specification is adopted to improve the image contrast and highlight the target information. Finally, the adaptive median filter and Wiener filter are used for denoising processing, which provides a good premise for the subsequent image segmentation. The effect before and after image denoising is shown in Figure 3.

The article "Manifestation of Urinary Tract Injury during Cervical Cancer Surgery Based on CT Urography Secretion Phase Images" was published in 2022. Journal: Contrast Media Mol Imaging.

## 3. Experimental Study on the Impact of Urinary Tract Injury during Cervical Cancer Surgery

### 3.1. Experimental Samples

A retrospective analysis of the clinical data of cervical cancer patients in the Obstetrics and Gynecology Department of the First Hospital of the city from March 2019 to October 2020. All cases included in the study underwent extensive total hysterectomy combined with pelvic lymph node dissection ± para-aortic lymph node dissection after preoperative evaluation. According to the different MIS adopted, the included patients will be grouped.

### 3.2. Sample Selection

#### 3.2.1. Inclusion Criteria

1. The pathological diagnosis of cervical cancer is clear
2. FIGO clinical staging (2009) is cervical cancer of stage IA-IIA
3. Patients with stage IIB cervical cancer who received radiotherapy and chemotherapy before surgery
4. Those who have normal heart function and lung function and can tolerate major surgery

#### 3.2.2. Exclusion Criteria

1. Malignant tumors of other systems
2. Patients with medical diseases that affect survival
3. Patients with metastatic tumors

The article "Manifestation of Urinary Tract Injury during Cervical Cancer Surgery Based on CT Urography Secretion Phase Images" was published in 2022. Journal: Contrast Media Mol Imaging.

### 3.3. Routine Preoperative Testing

1. Ask the patient's general condition and past medical history in detail, understand the patient's general health status, and clarify the surgical indications and whether there are surgical contraindications;
2. Actively improve relevant preoperative examinations, such as blood routine, liver and kidney function, electrolytes, blood sugar, blood type, urine routine, stool routine, blood coagulation series, preoperative infection, electrocardiogram, and chest X-ray;
3. Routine gynecological examinations and cervical exfoliative cytology examinations include human papillomavirus (HPV) and liquid-based cytologic test (thinprep cytologic test, TCT), gynecological pelvic ultrasound, hepatobiliary pancreatic spleen ultrasound, urinary system ultrasound, and pelvic MRI (magnetic resonance imaging);
4. Elderly patients or patients suspected of having cardiopulmonary function abnormalities need to undergo heart and lung function tests and both lower extremity venous thrombosis tests if necessary. Cardiac ultrasound and pulmonary function tests are used to assess whether the patient's heart and lung functions can withstand major operations with head low buttocks high; ultrasound of the veins of both lower extremities is used to rule out whether the patient has peripheral vascular disease.

### 3.4. Preparation before Surgery

1. Routine abdomen cleaning and perineal skin preparation;
2. Prepare the vagina and intestines as usual before surgery;
3. Routinely prohibit patients from eating and drinking 8–12 hours before surgery, and prohibit patients from drinking water within 4–6 hours before surgery;
4. It is recommended that patients wear elastic stockings correctly during and after the operation, which can prevent venous thrombosis of the lower extremities.

### 3.5. Statistical Methods

All relevant data are analyzed using SPSS 24.0 statistical software. The results of numerical variables are expressed as the mean standard deviation (*x*, *s*), and categorical variables are expressed as frequency and percentage. For the numerical variables that meet the uniformity and the regularity of change at the same time, the analysis of the change is selected for comparison between groups. For categorical and numerical variables that cannot satisfy the uniformity and normality of variation at the same time, nonparametric tests should be selected. Chi-squared test was used for comparison between groups. If *P* < 0.05, the difference is considered statistically significant.

## 4. Experimental Analysis of the Impact of Urinary Tract Injury during Cervical Cancer Surgery

### 4.1. Basic Clinical Indicators of Patients

Table 2 shows the general clinical data of patients in the nano-drug-loaded surgery group and laparoscopic surgery group, and Table 3 shows the number of different pathological types.

The article "Manifestation of Urinary Tract Injury during Cervical Cancer Surgery Based on CT Urography Secretion Phase Images" was published in 2022. Journal: Contrast Media Mol Imaging.

A total of 494 patients with cervical cancer were included in this study. According to different surgical methods, they were divided into a nano-drug-loaded surgery group and a laparoscopic surgery group. Among them, there were 368 cervical cancer patients in the nano-drug-loaded surgery group. The average age of cervical cancer patients in the nano-drug-loaded group was 45.78 ± 8.72 years, and their average body mass index BMI was 21.63 ± 3.91.

In the laparoscopic surgery group, 56 patients had a history of pelvic and abdominal surgery. The patients in the study period had received radiotherapy and chemotherapy before surgery. After the tumor size was reduced, the patients underwent surgical treatment after being evaluated by two experts above the subtropical height.

It can be seen from the table that there was no statistically significant difference between the two groups of patients in terms of age, FIGO staging, pathological type, and pelvic and abdominal surgery history (*P* > 0.05). The average BMI of the nano-drug-loaded surgery group was larger than that of the laparoscopic surgery group, and the difference was statistically significant (*p*=0.022).

All operations of the patients in the nano-drug-loaded surgery group were successfully performed, and no case was converted to laparotomy. The OT of the patients in the nano-drug-loaded surgery group was 195.00 (167.50, 225.00) min, and the EBL was 50 (30, 50) ml. No patient required blood transfusion. The average number of lymph nodes dissected during the operation was 18 (15, 24). The details are shown in Table 4.

It can be seen from the table that the OT of the patients in the laparoscopic surgery group is 170.00 (152.50, 200.00) min, the EBL is 100 (50, 200) ml, and the average number of lymph nodes dissected during the operation is 18 (15, 23). One patient in the laparoscopic surgery group received 1400 ml of intraoperative bleeding and was infused with 4 U of red blood cells and 350 ml of plasma.

### 4.2. Comparison of Postoperative Scores

Among the surgical patients included in the study, except for one patient with cervical cancer who was originally planned to undergo laparoscopic surgery because of severe pelvic adhesions and unable to successfully establish a pneumoperitoneum, the surgery was successfully completed for the rest of the patients. We made statistics on whether these patients had postoperative complications, as shown in Figure 4.

In the nanomedicine surgery group, there were 13 cases of urinary retention, 3 cases of lymphatic cysts, and 2 cases of postoperative colon failure. The infections were cured after local treatment. Four cases of hydronephrosis occurred after the operation, a renal tubule “J” was implanted in the patient with hydronephrosis, and a renal tubule “J” was implanted in the right kidney of another patient with hydronephrosis, and 2 cases of venous thrombosis of the lower extremities. In the laparoscopic surgery group, 8 cases had urinary retention, 4 cases had lymphatic cysts, 1 case had vaginal colitis after operation, and 3 cases had pelvic abscess after operation. All recovered after combined anti-infective treatment. One patient received bladder syringe treatment due to poor recovery of bladder function after surgery. Two patients had a syringe for urinary tract and repair after surgery. Hydronephrosis occurred in 3 cases, and hydronephrosis occurred in 1 case. The “J” tubes of both kidneys are inserted through lower limbs. It can be seen from Figure 3 that 6.50% of the patients in the nanomedicine surgery team had postoperative complications, which was lower than the incidence of postoperative complications in the laparoscopic surgery group (19.20%) with significant difference (*P* < 0001).

The article "Manifestation of Urinary Tract Injury during Cervical Cancer Surgery Based on CT Urography Secretion Phase Images" was published in 2022. Journal: Contrast Media Mol Imaging.

We statistics the postoperative pathological data of patients, and compare the postoperative conditions of patients between different methods, as shown in Figure 5.

LL—cervical interstitial infiltration depth <0.5 cm; LS—cervical interstitial infiltration depth ≥0.5 cm; PP—parauterine infiltration positive; PL—parauterine infiltration negative; VP—vascular infiltration positive; VN—vascular infiltration negative; LP—pelvic lymph node metastasis is positive; LN—pelvic lymph node metastasis is negative.

From the image, there are 12 cases (31,58%) in the observation group with a cervical infiltration depth of 0,5 cm, and 47 cases (94,00%) in the control group. The difference was statistically significant (*P* < 0001). Note: no patients in the control group were filtered for neutrophils, and 3 patients (6,00%) in the control group were filtered for neutrophils. There was no significant difference (*P*=0345). There were 0 cases of lymphatic infiltration in the observation group (0,00%) and 7 cases of lymphatic infiltration in the control group (14,000%). The difference was statistically significant (*P*=0,045) in 2 cases of lymph node metastasis in the observation group (5,30%) and 14 cases of lymph node metastasis in the control group (28,00%). The difference was statistically significant (*P*=0006).

After the treatment, we monitored the patient. The average monitoring time is 29 months, the longest monitoring time is 17 months, and the shortest monitoring time is 44 months. Of the 38 cases in the observation group, 3 cases were lost to follow-up, 7 cases were lost to follow-up, and 50 cases in the control group were lost to follow-up. The rate of loss to follow-up was 8.00%. The detailed information is shown in Figure 6.

The article "Manifestation of Urinary Tract Injury during Cervical Cancer Surgery Based on CT Urography Secretion Phase Images" was published in 2022. Journal: Contrast Media Mol Imaging.

From the image, during the monitoring period, there were 5 relapses in the observation group without death. There were 7 recurrences in the control group, of which 1 patient died of recurrence due to failure to add radiotherapy 23 months after surgery, and 2 patients died after recurrence at 15 months and 21 months after surgery. Figure 2 shows the survival curves of patients in the observation group and the control group. The 3-year overall survival rates of the observation group and the control group were 100,00% and 92,80%, respectively, with no significant difference (*P*=0,20).

### 4.3. Postoperative Quality of Life of Patients

A total of 81 patients with cervical cancer were followed up in this study, and 3 cases died. There were 56 cases who completed the QOL-UCC Quality of Life Evaluation Scale. Among them, 19 patients in the observation group filled out the scale completely, and 37 patients in the control group filled out the scale completely. The specific situation is shown in Figure 7.

Group A evaluated the physical health of the patients, including 7 items including abnormal vaginal bleeding, leucorrhea changes, lower abdomen or waist or lower limb pain, appetite, mental status, fatigue time, and sleep status. The observation group score was 4.57 (4.43, 4.71) points; the control group score was 4.71 (4.43, 4.79) points. Group B evaluated the patient's mental health from five aspects: mood, anxiety, depression, low self-esteem, and self-perception differences. The observation group score was 4.40 (4.00, 4.90) points, and the control group score was 4.80 (3.80, 4.90) points. Group C evaluates the performance of patients' social functions, including daily self-care status, work status, housework status, getting along with the surrounding people, the frequency of postoperative intercourse, the degree of satisfaction with sex life, and whether they get along well with their spouses. The observation group scored 3.17 (2.67, 3.71) points, and the control group scored 2.86 (2.57, 3.28) points. Group D mainly analyzes the patients' expectations and interests in survival, whether they are willing to participate in leisure and entertainment activities, and whether there is any change in their hopes and plans for long-term life. The observation group score was 3.33 (3.00, 4.00) points, and the control group score was 4.00 (3.67, 4.17) points. Group E evaluates the negative effects of treatment, including the impact of radiotherapy on urination, the degree of family economic status and menopausal symptoms. The observation group score was 3.67 (3.00, 4.50) points, and the control group score was 3.67 (3.00, 4.00) points.

The article "Manifestation of Urinary Tract Injury during Cervical Cancer Surgery Based on CT Urography Secretion Phase Images" was published in 2022. Journal: Contrast Media Mol Imaging.

We conducted a statistical survey on whether patients can be integrated into their daily lives, as shown in Figure 8.

It can be seen from Figure 8 that the patients who used the nanodrug delivery system surgery in this article are better integrated after the operation. The two groups of patients have no obvious five aspects of physical health, mental health, social function performance, survival expectations and interests, and the negative effects of treatment with significant difference (*P* > 0.05).

The pathological types of cervical cancer are mainly divided into squamous cell carcinoma, adenocarcinoma, adenosquamous carcinoma, and other types such as neuroendocrine carcinoma. The nanodrug delivery system group, the laparoscopic group, and the laparotomy group each have a patient with a special pathological type, namely, small cell carcinoma, clear cell carcinoma, and small cell carcinoma. The overall pathological types of the three groups were similar in distribution. The postoperative pathological results of the three groups of patients are shown in Figure 9.

The postoperative pathological results of the three groups of patients are shown in Figure 9. Positive lymph nodes, positive parauterine tissues, or positive surgical margins are high-risk factors for cervical cancer recurrence. Those who have any of the above require additional postoperative radiotherapy. The distribution of these three high-risk factors in the three groups of patients was similar. The *P* values are all greater than 0.05.

## 5. Conclusion

The article shows that the nanodrug delivery system can reduce the volume of local tumor lesions, reduce the clinical stage of the tumor, and bring more surgical treatment opportunities for patients with locally advanced cervical cancer. In addition, pelvic lymph node metastasis and the median depth of the cervix are important factors affecting the clinical prognosis of patients. The postoperative pathological diagnosis results of the two groups were compared. The depth of cervical filtration, vascular filtration rate, and lymph node metastasis rate in the observation group were lower than those in the control group (*r* < 0.05). The above results indicate that the nanodrug distribution system may affect the clinical efficacy of cervical cancer patients. Of course, this article also has some shortcomings. When this study summarizes the results of clinical problems, the relevant research evidence included is less and of poor quality, and there is a lack of high-quality research. Therefore, in future research, we consider including high-quality original research through various channels in order to better confirm the conclusions of this research. Due to the short production cycle and lack of corresponding conditions (time, funds, manpower, and other resources), this study has not organized an expert consensus meeting of the guideline group to discuss the degree of conformity between the evidence and the clinical issues, and did not invite experts to modify the opinions of the issues that have been raised. No complete and effective recommendations have been formed. Therefore, we will supplement the members of the guideline group when conducting follow-up research on the full version of the guideline, and make more adequate plans for future research.

The article "Manifestation of Urinary Tract Injury during Cervical Cancer Surgery Based on CT Urography Secretion Phase Images" was published in 2022. Journal: Contrast Media Mol Imaging.

## Figures and Tables

**Figure 1:** Schematic diagram of the drug delivery system.

**Figure 2:** The treatment process.

**Figure 3:** Image denoising effect.

**Figure 4:** Postoperative complications.

**Figure 5:** Postoperative pathology.

**Figure 6:** Follow-up of patients.

**Figure 7:** Postoperative quality of life.

**Figure 8:** Daily life survey of patients.

**Figure 9:** Pathological results between groups.

**Table 1:** Cervical cancer staging.

FIGO staging	Tumor area
I	Stage I tumors are limited to the uterus
I A	Invasive cervical cancer diagnosed under microscope
II	The tumor exceeds the cervix and does not reach the pelvic wall
II A	Tumor does not invade parauterine tissues
III	The tumor reaches the pelvic wall or 1/3 of the vagina
III A	The tumor invaded the lower 1/3 of the vagina without invading the pelvic wall
IV	Tumor invades the bladder or rectal mucosa
IV A	Tumor dissemination value adjacent organs
IV B	Distant metastasis of tumor

**Table 2:** General clinical data of patients.

	Nano-drug-loaded surgery group	Laparoscopic surgery group	*T*/*x*^2^	*P*
Total number (cases)	368	124	—	—
Age	45.78 ± 8.72	45.82 ± 8.02	−0.045	0.954
BMI	21.63 ± 3.91	20.82 ± 3.17	2.301	0.021
Staging (example)	—	—	3.486	0.511
I	32	2	—	—
I a	205	78	—	—
II	98	22	—	—
II a	34	22	—	—

**Table 3:** The number of people with different pathological types.

Pathological type	Nano-drug-loaded surgery group	Laparoscopic surgery group	*T*/*x*^2^	*P*
Squamous cell carcinoma	323	111	—	—
Adenocarcinoma	25	8	—	—
Other	10	6	—	—
History of pelvic and abdominal surgery	181	56	0.752	0.373

**Table 4:** Postoperative conditions of patients.

	Nano-drug-loaded surgery group	Laparoscopic surgery group	*T*/*x*^2^	*P*
Operation time (min)	184	169	5.049	<0.001
Intraoperative blood loss (ML)	50	100	−5.114	<0.001
Intraoperative blood transfusion	0	1	0.313	0.569
Conversion to laparotomy	0	1	0.313	0.569
Exhaust time (d)	1.29 ± 0.21	1.42 ± 0.22	−1.554	0.043
Maximum body temperature (°C)	14	20	−4.123	<0.001
Maximum body temperature (°C)	37.5	37.6	−1.780	0.049
Length of stay (d)	6	6	−2.693	0.007
Number of lymph node dissections	18	18	0.368	0.605

The article "Manifestation of Urinary Tract Injury during Cervical Cancer Surgery Based on CT Urography Secretion Phase Images" was published in 2022. Journal: Contrast Media Mol Imaging.

## Data Availability

The datasets used or analyzed during the current study are available from the corresponding author on reasonable request.
